The article "A Human-Machine Interface Based on an EOG and a Gyroscope for Humanoid Robot Control and Its Application to Home Services" was published in 2022. Journal: J Healthc Eng.

# A Human-Machine Interface Based on an EOG and a Gyroscope for Humanoid Robot Control and Its Application to Home Services

**DOI:** 10.1155/2022/1650387

**Published:** 2022-03-19

**Authors:** Fan Wang, Xiongzi Li, Jiahui Pan

**Affiliations:** ^1^School of Software, South China Normal University, Guangzhou 510631, China; ^2^Engineering Research Center for Intelligent Robotics, Ji Hua Laboratory, Foshan 528200, China

## Abstract

The human-machine interface (HMI) has been studied for robot teleoperation with the aim of empowering people who experience motor disabilities to increase their interaction with the physical environment. The challenge of an HMI for robot control is to rapidly, accurately, and sufficiently produce control commands. In this paper, an asynchronous HMI based on an electrooculogram (EOG) and a gyroscope is proposed using two self-paced and endogenous features, double blink and head rotation. By designing the multilevel graphical user interface (GUI), the user can rotate his head to move the cursor of the GUI and create a double blink to trigger the button in the interface. The proposed HMI is able to supply sufficient commands at the same time with high accuracy (ACC) and low response time (RT). In the trigger task of sixteen healthy subjects, the target was clicked from 20 options with ACC of 99.2% and RT 2.34 s. Furthermore, a continuous strategy that uses motion start and motion stop commands to create a certain robot motion is proposed to control a humanoid robot based on the HMI. It avoids the situation that combines some commands to achieve one motion or converts the certain motion to a command directly. In the home service experiment, all subjects operated a humanoid robot changing the state of a switch, grasping a key, and putting it into a box. The time ratio between HMI control and manual control was 1.22, and the number of commands ratio was 1.18. The results demonstrated that the continuous strategy and proposed HMI can improve performance in humanoid robot control.

## 1. Introduction

Humanoid robots, resembling the human body in terms of shape and range of actions, can replace individuals in performing daily home tasks such as grasping, lifting objects, and turning on/off switches of electrical equipment. HMI is able to translate human intentions into external device control commands, helping people perform certain daily tasks with the help of a robot. There is much research concentrating on HMIs for robot control, such as joysticks [1] and keyboards [2]. However, these manual interfaces become useless for persons suffering from severe neuromuscular disorders caused by an accident or congenital disease. With modern life-support technology, paralyzed people can lead lives that are enjoyable and productive if they can be provided with novel nonmanual means of communication and control [3].

The article "A Human-Machine Interface Based on an EOG and a Gyroscope for Humanoid Robot Control and Its Application to Home Services" was published in 2022. Journal: J Healthc Eng.

A major task of designing a nonmanual HMI for humanoid control is to rapidly, accurately, and sufficiently produce commands to perform some daily tasks as people do [4], including navigation control, such as left/right turn, forward and backward, and some joint control. Since many paralyzed people maintain normal head and eye function, electroencephalogram (EEG) or EOG, resulting from brain activity and eye movement, respectively, can be used in HMIs and have attracted a great deal of attention over the past few decades [5]. EEG and EOG have merits because they are noninvasive, technically less demanding, and widely available at relatively low cost.

An EEG-based HMI is a type of brain computer interface (BCI) that conveys a user's intent via brain signals that do not depend on neuromuscular activity. Common EEG patterns used in BCIs include event-related potentials (ERPs, e.g., the P300 potential [6]), the mu/beta rhythm related to motor imagery (MI [7]), and steady-state visually evoked potentials (SSVEPs [8]). Several BCIs aimed at controlling robotic humanoids have been reported [9–11]. Spataro et al. proposed a P300-based BCI to actuate a humanoid robot to fetch a glass of water [9], with subjects using the P300 signal to choose a highlighted grid in a user interface. The accuracy of the system was 74.5%. In [10], Saduanov et al. developed a framework for a P300-based BCI telepresence robot. The robot can execute 16 commands, including 7 present commands and 9 navigation commands. The real-time accuracy of the robot was above 78% on average. A 6-command SSVEP-NAO robot system was developed in [11]. The online experimental results of the system showed that it yielded an average accuracy of 83.5%. To our knowledge, EEG-based HMIs for humanoid robotic control typically implement P300 and SSVEP paradigms to control a device due to their sufficient commands. However, the disadvantage of these paradigms is that accuracy and response time are limited by the number of commands. The more commands a system has, the more targets the BCI paradigm has. Increasing the number of targets makes a P300 paradigm have a longer round time, while a system using an SSVEP paradigm needs additional different frequency signals for identification [12]. Therefore, for the P300 paradigm, the designer needs to trade off sufficient commands and low RT; for the SSVEP paradigm, ACC and sufficient commands should be carefully weighed.

An EOG signal has also been used to design nonmanual HMIs. Typical eye movements include gaze, blink, wink, and frown. All of these movements can generate prominent EOG features with high signal-to-noise ratios (SNRs). Therefore, some studies have constructed EOG-based HMIs to control external devices. In [13], Ameri proposed an imperceptible EOG sensor system to control a quadcopter via eyeball movement (left, right, up, down, and blink). The five eye movements were directly translated into five control commands (right, left, up, down, and straight) to control the quadcopter. In 2020, Milanizadeh and Safaie used the subject's eye movement toward the four middle parts of the screen edges of a laptop to navigate quadcopter with a 0.6 s delay and an accuracy of 94.8% [14]. In 2021, Triadi et al. constructed a mouse control system using eight eye movements to control the cursor's movement, including up, top right, top left bottom, bottom right, bottom left, right, and left. The RT and ACC of the system in a customized dataset were 1.97 s and 100%, respectively [15]. An EOG-based HMI for wheelchair control was proposed in Huang and He's research. The system provided a GUI with 13 flashing buttons that correspond to 13 wheelchair commands (navigation, speed control, and stopping commands). The user issued a command by blinking according to a button's flashes. The system achieved an average EOG accuracy of 96.7% and an RT of 3.53 s [5]. In the case of the IoT platform based on EOG, Molleapaza-Huanaco et al. used three saccadic movements of the eye to encode eight control commands of wheelchairs, obtaining a classification accuracy rate of 93% [16]. Sharma et al. proposed an EOG-based HMI for robotic arm control by detecting a user's eye closing/opening and eye blinks [17]. The system can issue 7 commands (left, right, up, down, forward, backward, and grip) with an accuracy of 96.9%. In summary, EOG-based HMI has two main implements: eye movements without an interface and blinks with an interface. The first implementation belongs to the asynchronous system, but it is subject to the number of eye movements without sufficient commands. Moreover, eyeball movement is a voluntary behavior, and the false trigger problem in the idle state still needs to be solved. In the second implementation, the interface ensures sufficient commands. Meanwhile, the flashed cue and blink trigger conditions make the false trigger decrease. However, these flashed paradigm systems are usually synchronous, and the RT is unsatisfactory for device control. Consequently, one main challenge still exists for EOG-based HMIs: constructing an asynchronous system providing sufficient commands with low RT.

The article "A Human-Machine Interface Based on an EOG and a Gyroscope for Humanoid Robot Control and Its Application to Home Services" was published in 2022. Journal: J Healthc Eng.

To overcome the limitations of existing systems, this paper proposes an EOG and gyroscope-based HMI for humanoid robot control. In our system, a multilevel GUI is designed to output sufficient robot control commands. Users use a double blink EOG and two-angle data provided from a gyroscope to generate a cursor clicking event. By triggering buttons at different levels, users can implement navigation or joint motion of a robot. Two online experiments with sixteen subjects were conducted. First, all of the subjects participated in a synchronous experiment in which they tested the proposed HMI by triggering the target buttons. Next, the subjects manipulated a humanoid robot using the proposed HMI to complete a home service task in a simulation environment (asynchronous experiment). Indicators, such as the accuracy, response time, and false positive rate, were calculated. The results demonstrated that the proposed asynchronous HMI based on only one type of eye movement (double blink) and two angular velocities could rapidly, accurately, and sufficiently produce commands to control a humanoid robot completing home service tasks.

## 2. Materials and Methods

### 2.1. Signal Acquisition

In this study, EOG signal and gyroscope data are collected by a device from HNNK Company, as shown in Figure 1. The sampling rate of the device was 125 Hz. Three electrodes (“CH1,” “COM,” and “COMLEG”) are attached to the skin, and the impedances between the skin and the three electrodes are kept below 5 kΩ. Among the three channels, “CH1” is the data channel to record vertical EOG signals from the forehead. The central position of the device has a gyroscope to detect the angular change of the gyroscope when the user rotates his head.

### 2.2. Graphical User Interface

The architecture of the GUI used in this study is illustrated in Figure 2. The main window consists of two panels: a navigation panel and a joint control panel. The navigation panel is consistent, including 8 navigation buttons and 3 speed control buttons (slow, general, and fast types for walking and joint rotation control), while the joint control panel changed from three levels: joint selection, joint motion selection, and stopping. The details of each level are described as follows.

- Joint selection level: nine buttons represent different joint objects, such as the head, LShoulder (left shoulder), LElbow (left elbow), etc.
- Joint motion selection level: two or four buttons represent motions of a certain joint, and one return button gives the opportunity to modify the chosen joint. The number of buttons at this level is determined by the joint that was chosen at the joint selection level. As shown in Figure 2, the motion selection level has 4 buttons to represent the two-axis rotations of the shoulder. Images in the middle of buttons illustrate positive (+) and negative (−) directions of certain axis motion.
- Stopping level: a large button stops a navigation or joint rotation motion.

The article "A Human-Machine Interface Based on an EOG and a Gyroscope for Humanoid Robot Control and Its Application to Home Services" was published in 2022. Journal: J Healthc Eng.

### 2.3. Control Mechanism

The proposed HMI combines an EOG signal and a gyroscope to realize a robot control system. As illustrated in Figure 3, the system consists of four parts: a signal acquisition device, a GUI display program, a signal processing program, and a humanoid robot. The acquisition device (HNNK device) collects the EOG and angular change data transmitted to the signal processing program for classification. If a button triggering event exists, the GUI display program will output a relevant command to the humanoid robot.

A button triggering event consists of two conditions: a double blink feature in the EOG signal and the cursor location in the GUI. As depicted in Figure 4, the collection device provides two types of data: an EOG signal and three angles of the gyroscope. We use the yaw angle and roll angle to control the cursor while detecting a double blink in the EOG signal. Users trigger a button when the cursor is on the button with a double blink.

In the command generation part, we propose a continuous control strategy. It disassembles each real motion of the robot into two phases: one phase that makes the robot continuously move or rotate and another phase that makes the current continuous motion stop. In the first phase, the user triggers a command for navigation or joint motion by clicking buttons with the GUI, making the robot start to move or rotate continuously. Then, the stop button is triggered at the right moment to make the robot stop at a desired position or pose in the second phase. The process of using this strategy to control the humanoid robot to implement navigation or joint motion is illustrated in Figure 5. Initially, a navigation control panel and a joint control panel are presented, and the joint selection level is presented in the joint control panel first. The user can select one button from the navigation control panel or joint control panel. If the navigation control button is selected, the robot will receive the relative command to move continuously. Meanwhile, the stopping level is presented in the joint control panel, and the navigation command buttons in the navigation panel are invalid. If the joint control button is selected, the joint motion selection level will be presented, and navigation commands will become unavailable. The user can choose to return to the joint selection level or rotate the current joint by clicking the button in joint control panel. When a motion is selected, the robot will rotate the joint to a certain direction continuously, and the joint control panel will present the stopping level. At the stopping level, users need to stop the current movement of the robot regardless of whether the movement is generated from the navigation panel or joint control panel.

The article "A Human-Machine Interface Based on an EOG and a Gyroscope for Humanoid Robot Control and Its Application to Home Services" was published in 2022. Journal: J Healthc Eng.

### 2.4. Algorithm

In this study, the algorithm can be divided into two parts: (i) cursor position calculation and (ii) double blink detection. The cursor position is derived from the angle data of the gyroscope. Double blink waveform detection is performed anytime in the EOG signal. First, a subsegment (duration of 1 s) is derived from 125 recorded EOG signal points, and the similarity between the subsegment and double blink segment generated in the threshold calculation part is calculated. When the subsegment is similar to the double blink segment, several features are extracted, such as the energy and duration of the blink. The algorithm determines whether these features satisfy the threshold conditions. A double blink exists in the subsegment if all the thresholds are met. Further details are described in the following paragraphs.

#### 2.4.1. Cursor Position Calculation

The HNNK device can provide three tilts (yaw, roll, and pitch) when the user rotates his head. The signal processing program saves the initial value of the three tilts when the user wears the device, and the center of the screen is set as the initial position of the cursor. A head rotation motion changes the three tilts, resulting in Δyaw, Δroll, and Δpitch related to the initial tilts. The program uses Δyaw and Δroll to calculate Δ*x* and Δ*y* of the cursor location based on the initial position. Then, Δ*x* and Δ*y* are used to update the position of the cursor in real time. The calculation formulas are as follows:

(1) $$\begin{array}{c} \left\{\begin{array}{c} \Delta x=\;\frac{\Delta \text{yaw}}{pi\;\times \;180}\times \left(1+s\right),\\ \Delta y=\frac{\Delta \text{roll}}{pi\times 180}\times \left(1+s\right),\\ x_{\text{new}}\;=\;x_{\text{initial}}\;+\;△x,\\ y_{\text{new}}\;=\;y_{\text{initial}}\;+\;△y, \end{array}\right. \end{array}$$

where (*x*_new_, *y*_new_) is the calculated position of the cursor and *s* is a factor to adjust the sensitivity of the cursor ranging from −0.5 to 0.5.

#### 2.4.2. Double Blink Detection

*(1) Preprocessing*. First, the signal processing program filters the recorded EOG signal through a digital bandpass filter (1–10 Hz) to remove high-frequency noise and eliminates the effect of baseline drift [18]. Then, a subsegment (duration is 1 s) is derived from 125 sampling points of the filtered EOG signal, and the similarity between it and the double blink segment is calculated. In this study, the Pearson correlation coefficient (PCC) is used to evaluate the similarity of the two signals (equation (2)). If the PCC is over the similarity threshold, the waveform features will be extracted. Otherwise, the subsegment does not exist a double blink segment.

(2) $$\begin{array}{c} \text{Cov}\left(x,y\right)=\frac{\sum_{i}^{N}\left(x_{i}-\bar{x}\right)\left(y_{i}-\bar{y}\right)}{N-1}, \end{array}$$

where *x* and *y* are vectors with *N* dimensions representing the two signals, *x*_*i*_/*y*_*i*_ represents the value of the *i* th dimension, and Cov(*x*, *y*) indicates the similarity of the two signals *x* and *y*, ranging from −1.0 to 1.0 [19].

*(2) Waveform Feature Extraction*. As shown in Figure 6, there are two visible peaks in the double blink waveform. Therefore, the program identifies the positions of these peaks to extract the features. Specifically, the extreme points corresponding to the maximum value and secondary maximum value are regarded as peak1 and peak2. Here, *t*_peak1_ and *t*_peak2_ are used to denote the positions of peak1 and peak2. Then, two features *d* and *e* are calculated as follows:

(3) $$\begin{array}{c} d=t_{\text{peak}2}-t_{\text{peak}1},\\ e=\overset{t=t_{\text{peak}2}}{\underset{t=t_{\text{peak}1}}{\sum }}x_{t}^{2}, \end{array}$$

where *d* and *e* represent the duration and energy between peak1 and peak2, respectively [20]. *x*_*t*_ is the voltage at the *t* th sampling point.

*(3) Double Blink Detection*. The program uses two duration thresholds *D*_min_ and *D*_max_ and two energy thresholds *E*_min_ and *E*_max_ to realize double blink waveform detection, as follows:

(4) $$\begin{array}{c} r=\left\{\begin{array}{cc} 1, & \text{if }D_{\min}\leq d\leq D_{\max}\text{ and }E_{\min}\leq e\leq E_{\max},\\ 0, & \text{otherwise,} \end{array}\right. \end{array}$$

where *r* is the result of double blink detection. Specifically, *r* = 1 indicates that a double blink is detected, whereas *r* = 0 indicates that no double blink is detected. The threshold parameters *D*_min_, *D*_max_, *E*_min_, and *E*_max_ in equation (4) are determined in a calibration process, which will be described later.

The article "A Human-Machine Interface Based on an EOG and a Gyroscope for Humanoid Robot Control and Its Application to Home Services" was published in 2022. Journal: J Healthc Eng.

#### 2.4.3. Threshold Calculation

The thresholds *D*_min_, *D*_max_, *E*_min_, and *E*_max_ and the double blink segment vary among individuals. Thus, a calibration process is performed for each user before he or she starts to use the EOG-based HMI. Specifically, a single button (“Blink”) is presented on the center of the screen, flashing 10 times with a 3 s duration. The user needs to generate a double blink according to each flash of the button. Similar to the blink detection process, the recorded EOG is filtered, and a subsegment is derived for each flash. Waveform features, including *d* and *e*, are extracted from these 10 subsegments. If the user misses one flash, the corresponding subsegment is removed, and the features are averaged across the rest of the subsegments. The duration thresholds *D*_min_ and *D*_max_ are the minimum and maximum of the *d* features in these subsegments. The energy thresholds *E*_min_ and *E*_max_ are calculated by multiplying the average value of *e* by empirical factors (*E*_min_ = 0.8 × $\;\bar{e}$ and *E*_max_ = 1.2 × $\bar{e}$). To obtain the double blink segment of a person, the subsegments are averaged to generate a representative segment.

## 3. Experiments and Results

To evaluate the performance of the proposed HMI for humanoid robot control, sixteen healthy subjects, aged 23 to 27, participated in two online experiments. All subjects had normal or corrected-to-normal vision. Before performing the experiments, each subject was instructed to read and complete an informed consent form. First, a calibration session was performed to determine the four thresholds and the double blink segment, as described in Section 2.4.3. Then, experiments were performed within one day for each subject with 10 min breaks between every two consecutive experiments.

### 3.1. Experiment I: Clicking Target Buttons

The proposed humanoid robot control system uses a continuous control strategy to perform a motion with two commands (a certain motion start command and a motion stop command). The experiment uses two subexperiments, a general button triggering task and a stop button triggering task, to evaluate the performances of the motion start command triggering and motion stop command triggering.

#### 3.1.1. General Button Click Experiment

In this experiment, subjects were asked to use the proposed HMI triggering button in the panel (Figure 7(a)), which is used to generate a navigation or joint motion command. Specifically, subjects were tasked with selecting randomly generated target buttons (target button flashed to let subjects know). The subject had 5 s to click the target after it flashed. In addition, there was an idle state, a random period in the range of 10∼20 s, between each pair of consecutive target triggering tasks. The random duration aimed to eliminate the subjective prediction influence of people [4]. Indicators, such as the ACC, RT, and FPR, were calculated using the experimental results. The entire experiment time was 5 min, and each subject finished the experiment five times. The rest time was 5 min between two consecutive experiments.

#### 3.1.2. Stop Button Click Experiment

This experiment aimed to evaluate the performance of stop motion command triggering in the control process because it directly influences the precision of navigation and joint control. In this experiment, the GUI had one large stop button, which was a unique target, and the other navigation buttons were unclicked, except the speed control buttons (Figure 7(b)). Subjects followed the prompt (flash) to click the stop button. Other things, such as the result metrics, experiment time, duration, and rest times, were identical to the general button clicked experiment.

The article "A Human-Machine Interface Based on an EOG and a Gyroscope for Humanoid Robot Control and Its Application to Home Services" was published in 2022. Journal: J Healthc Eng.

Table 1 illustrates the ACC, RT, and FPR for all subjects in the general button triggering task. On average, the subjects took 2.34 s to trigger a target button with 99.2% accuracy in the control state and produced a 0.34 event/min FPR in the idle state. In [21], the ACC, RT, and FPR of HMI-based motor imagery were 86.2%, 3.15 s, and 3.67/min, respectively. The proposed HMI has better performance. Compared with the EOG-based HMI for wheelchair control presented in [5] with an ACC of 96.7%, RT of 3.53, and FPR of 0 event/min, our HMI has a higher ACC and lower RT. The lower FPR of the EOG-based HMI is attributed to using a brain switch to achieve an asynchronous system. However, the solution determines that the switch between the work state and idle state of their system is less flexible than our proposed system and leads to a higher RT in command output. In a wheelchair control scenario, the FPR is more important, but the RT is more significant in a home service scenario.

The results in Table 2 show the performance of the stop button triggering task. The RT in this task was shorter than that in the general button triggering task because we used a large stop button, which made it easy to locate the cursor on the target. With decreasing RT, the ACC decreased from 99.3% to 97.4%, and the FPR increased to 0.74 events/min. The compromise suggests that users could send stop commands to terminate the robot's continuous movements immediately, which ensures that the robot performs the motion the person wants. It provides a solution for people who want to apply the proposed HMI to other scenarios with higher real-time requirements.

### 3.2. Experiment II: Humanoid Robot Control for Home Services

In Experiment II, the proposed HMI was used to control the navigation and joint motion of a humanoid robot (Nao H25, Softbank Inc., Japan, 0.573 m × 0.311 m) to complete a home service task, including an electric switch state change and an object grasping and placing. The default robot speeds of walking, turn direction, and joint rotation were set to 0.1 m/s, 0.39 rad/s, and 0.30 rad/s, respectively, which are the same as the general mode speed in the speed control function. We use a simulation environment from the 2014 Nao Challenge contest from Aldebaran Robotics and a virtual Nao robot in Webots 2021b (Figure 8). In the simulation environment for home service (a 9 m × 5 m room), the subject was instructed to control the robot from an initial position (position 1) to the switch position (position 2), turn on the switch, then go to the key position (position 3), grasp the key to the door, place the key in a pot (position 4), and rest at position 5. After finishing these tasks, the performance of each subject using the proposed HMI was recorded using metrics such as the information transfer rate (ITR), RT, ACC, and FPR. Different from the target button triggering experiment, all metrics have new meanings as follows.

(1) RT: the response time of robot command triggering. It is calculated according to
  (5) $$\begin{array}{c} \text{RT}=\frac{3\times {\text{RT}}_{g}\times N_{\text{joint}}+{\text{RT}}_{g}\times N_{\text{nav}}+{\text{RT}}_{s}\times N_{\text{stop}}}{N_{\text{joint}}+N_{\text{nav}}+N_{\text{stop}}}, \end{array}$$
  where RT_*g*_ and RT_*s*_ are the mean RTs of the general button trigger task and stopping button trigger task, respectively, and *N*_joint_, *N*_nav_, and *N*_stop_ are the quantities of joint control commands, navigation commands, and stopping commands in the experiments. Because joint control commands, unlike others, need two triggers of a general button in the joint control panel, with regard to the time the person chooses the second target button in the joint control command triggering, we use the three RTs of the general button to represent the RTs of joint control commands. The RT of the general button and the RT of the stop button represent the RT of navigation commands and the RT of the stop command, respectively.
(2) ACC: the possibility of a correct control command.
(3) FPR: false commands generated per minute during idle time.
(4) ITR: the bits of information transferred per minute, calculated according to
  (6) $$\begin{array}{c} \text{ITR}=\frac{60}{T}\times \left(\log_{2}\left(N\right)+P\times \;\log_{2}\left(P\right)+\left(1-P\right)\times \;\log_{2}\left(\frac{1-P}{N-1}\right)\right), \end{array}$$

where *N* is the number of commands, *P* is the average ACC, and *T* is the average RT.

The article "A Human-Machine Interface Based on an EOG and a Gyroscope for Humanoid Robot Control and Its Application to Home Services" was published in 2022. Journal: J Healthc Eng.

To further evaluate the controllability of the proposed HMI for humanoid robot control in home service, we designed a manual experiment in which each subject uses a physical mouse clicking the GUI button to control the robot to finish the tasks as a contrast test [21]. Similar to Experiment II, the EOG control and physical cursor control experiments were completed five times for each subject, and the average interval and commands of the five experiments are calculated.

The results of robot control in the home service scenario are shown in Table 3. The average accuracy was 99.3% across all subjects, resulting in an average ITR of 113.9 bits/min. Furthermore, each subject was able to complete the experiment 5 times without failure. These results demonstrate that the proposed continuous control strategy is valid to control a humanoid robot implementing navigation and joint motion in a home service task. The ACC of the real-time robot control is higher than that of the target button trigger experiment. The performance improvement could be mainly attributed to the fact that subjects were focused in the real-time control experiment without more double blinks because each command subjects sent had a real intention, making the robot navigate to a position or rotate a certain joint to a pose. True intention with a longer time makes subjects concentrate on the robot control process, which easily keeps subjects in a natural state [22,23]. In contrast, in the target button triggering experiment, each trial had a short and relatively fixed time. These truths cause fewer error commands in real-time robot control, leading to a higher accuracy and a lower FPR.

To investigate how similar the proposed HMI control performance was to manual control, we recorded the completion time and total number of commands of each subject in the operations of the humanoid robot and calculated the ratio of the measures in the two conditions (HMI control and manual control) shown in Figures 9 and 10. The time ratio between the proposed HMI control and the manual control was 1.22 on average, and the ratio of the number of commands was 1.18. In Jiang et al. [24], the time ratio and number of commands ratio were 1.49 and 1.53, respectively, in a 3DOF mobile robot arm control using a six-class BCI. Chae et al. also reported a time ratio of 1.27 in a robot navigation experiment using a three-class BCI [25]. Our result was better than these research results because the proposed HMI is an asynchronous system with a shorter command generation RT and the continuous control strategy that generates a realistic robot motion via only two commands, which means that the proposed HMI can save time and number of commands in a series of repeat commands in discrete control HMI. Furthermore, for complicated humanoid robot navigation and joint control, the reference experiment uses the same control GUI, which bridges the gap between the proposed HMI control and manual control.

## 4. Discussion

In this paper, we propose an HMI based on an EOG and a gyroscope that provides 40 control commands, including 8 navigation commands, 28 joint motion commands, 3 speed control commands, and 1 stopping command. A target triggering experiment suggests that the proposed HMI has a high accuracy and a short response time. The results of an asynchronous humanoid robot control indoor task demonstrated that the proposed HMI can efficiently control a humanoid robot to perform some daily home service tasks.

The article "A Human-Machine Interface Based on an EOG and a Gyroscope for Humanoid Robot Control and Its Application to Home Services" was published in 2022. Journal: J Healthc Eng.

For robot control, one challenge of HMIs is constructing an asynchronous system providing sufficient commands with low RT. In the proposed HMI, we use two self-paced and endogenous features, double blink and head rotation, to trigger the target. Self-space features make the HMI a natural asynchronous system, which means that users are able to select a command at their own convenience. It does not have a fixed interval in command output compared with a visually evoked potential HMI [26]. Therefore, the RT of the trigger is lower than most P300 and SSVEP HMIs and some EOG-based HMIs. Moreover, the double blink feature is detected using a single EOG signal. An EOG has a higher SNR than an EEG, and the double blink feature has a special waveform, which makes the double blink feature have a higher ACC than EEG features [27]. The higher ACC of the double blink and the condition of cursor position make the proposed HMI have an average accuracy of 99.3% in the robot control task.

Another challenge for robot control is that an HMI needs to output sufficient commands to support robots performing complicated tasks. For most visually evoked potential-based HMIs, increasing the target number of the GUI to support more commands increases the RT. Fortunately, some researchers have realized the problem of this solution, and they use a multilevel GUI to decrease the expression on RT, such as in [28,29]. However, another question results in the direction of navigation or joint rotation. These studies give only 3 to 5 commands, and other feasible motions of navigation or joint rotation cannot be represented. If a small step is used to represent them, a realistic robot motion will require a series of steps to achieve the goal, which means a series of repeated commands and increasing time, as in [30]. A continuous control strategy can solve this challenge. It sends a command to make the robot continuously move in a certain navigation or joint motion direction and then sends a stop command when a person considers the robot to be at the desired position or pose. Only two commands are needed to make the robot perform the desired motion. Of course, the continuous strategy has the shortcoming that users need to seize the right time to make the robot stop moving to control the robot movement accurately. The proposed system tackles it from two aspects. One is to reduce the response time by designing a large stop command to satisfy the triggering condition, easily decreasing the RT, and the other is to increase the speed control function, which allows users to control robot motion at different speeds (slow, general, and fast). Slower continuous movement is easy to stop, which creates more accurate motion. In the humanoid robot control experiment, all subjects finished the experiment without failure, and the average command ratio between the HMI control and manual control was 1.18, which demonstrates that our HMI system can efficiently accomplish some home service tasks with a higher requirement for control precision.

The article "A Human-Machine Interface Based on an EOG and a Gyroscope for Humanoid Robot Control and Its Application to Home Services" was published in 2022. Journal: J Healthc Eng.

There are also some limitations in the current work. First, the subjects needed to obtain more visual feedback information other than the robot's monocular vision when they controlled the robot to perform the daily home tasks. Such information roughly provided the positional relationship between the robot's arm and the object. In real life, a subject could obtain this visual information only when the robot was nearby. Second, subjects could not ensure accurate positional relationships from the visual information, unlike machine vision. Apart from this, the HMI control and automatic control were incomparable in object manipulation because the machine automatic control process could make full use of the location relationship data to calculate the appropriate trajectory for the robot's arm motion [31]. Motion planning of the arm will reduce the time used to control the arm manipulation of an object. We will try to do some work in the future to implement an automatic grasp system based on machine vision guidance and combine it with HMI control to implement a shared control system for humanoid robots [32]. This system will use HMI control to navigate the humanoid robot and determine the object that needs to be manipulated. Machine vision guidance control aims to automatically manipulate objects, which reduces the complexity and time of HMI control and increases the control precision [33]. With machine vision and HMI control, a person can use the humanoid robot system control to efficiently play a role in home service.

## 5. Conclusions

In this study, an EOG and a gyroscope-based HMI were developed to control a humanoid robot to perform home services. In our approach, a multilevel GUI was designed to supply sufficient commands controlling the humanoid robot. The subject wore a wireless collection device and used double blink and head rotation to trigger the button in the GUI. Different buttons responded to different commands, which enabled the subject to send commands by clicking buttons. Meanwhile, a continuous control strategy was proposed, which allowed the user to send an initial command to start the continuous motion of the robot and then send a second command to make the robot stop moving, performing the desired motion of the robot. The results of two online experiments demonstrated that the proposed HMI and continuous control strategy can be used to create an efficient humanoid robot control system for home service. In future work, we will reduce the FPR of the robot control system from two aspects: an EOG detection algorithm and continuous control strategy implementation.

The article "A Human-Machine Interface Based on an EOG and a Gyroscope for Humanoid Robot Control and Its Application to Home Services" was published in 2022. Journal: J Healthc Eng.

## Figures and Tables

**Figure 1:** HNNK device (location of three electrodes and a gyroscope for data recording).

**Figure 2:** The architecture of the proposed HMI GUI (the navigation panel is constant, but the content of the joint control panel is one of the levels).

**Figure 3:** Schema of the humanoid robot control system based on the proposed HMI.

**Figure 4:** Issuing a button click with the proposed HMI.

**Figure 5:** A continuous control strategy and a GUI are used to create a robot motion (the orange area and purple area are clickable panels).

**Figure 6:** The row EOG signal of double blink.

**Figure 7:** GUI of the button clicked experiment (robot in fast speed mode with gray background, so the fast button is unavailable): (a) general button click experiment GUI; (b) stop button click experiment GUI (blue button indicates the flashed button).

**Figure 8:** Top-down view of the humanoid robot control experiment environment.

**Figure 9:** The completion time for each subject in the home service task by proposed HMI control (blue bar) and manual control (gray bar). Avg indicates the average result of all subjects. The values above all subjects represent the time ratio of the proposed HMI control to the manual control.

**Figure 10:** The number of commands executed by the humanoid robot for each subject in the home service task via proposed HMI control (orange bar) and manual control (yellow bar). Avg indicates the average result of all subjects. The values above all subjects represent the command number ratio of the proposed HMI control to the manual control.

**Table 1:** The results of the general button triggering experiment.

Subject	RT (s)	ACC (%)	FPR (event/min)
S1	2.27	99.3	0.19
S2	2.24	98.5	0.41
S3	2.36	98.1	0.57
S4	2.33	98.8	0.43
S5	2.51	99.6	0.35
S6	2.24	99.7	0.38
S7	2.20	99.2	0.00
S8	2.58	99.4	0.27
S9	2.27	99.8	0.33
S10	2.24	99.5	0.31
S11	2.36	99.6	0.32
S12	2.33	99.2	0.24
S13	2.51	99.7	0.34
S14	2.24	99.4	0.42
S15	2.20	98.9	0.38
S16	2.58	98.6	0.51
Average	2.34	99.2	0.34

The article "A Human-Machine Interface Based on an EOG and a Gyroscope for Humanoid Robot Control and Its Application to Home Services" was published in 2022. Journal: J Healthc Eng.

**Table 2:** The results of the stop button click experiment.

Subject	RT (s)	ACC (%)	FPR (event/min)
S1	1.65	98.1	0.31
S2	1.23	95.6	1.41
S3	1.14	95.3	1.83
S4	1.27	97.8	1.12
S5	1.63	97.5	0.55
S6	1.51	98.7	0.39
S7	1.48	98.2	0.24
S8	1.35	96.4	0.47
S9	1.15	96.4	0.83
S10	1.39	98.3	0.26
S11	1.47	97.4	0.38
S12	1.31	96.7	0.64
S13	1.29	97.1	0.85
S14	1.62	98.9	0.59
S15	1.37	97.3	1.21
S16	1.43	98.8	0.69
Average	1.39	97.4	0.74

**Table 3:** The performance metrics of the proposed HMI during the humanoid robot control experiment.

Subject	RT (s)	ACC (%)	FPR (event/min)	ITR (bit/min)
S1	2.82	99.5	0.21	111.6
S2	2.68	99.4	0.28	117.2
S3	2.59	99.2	0.36	120.0
S4	2.58	99.5	0.29	122.3
S5	3.10	99.1	0.51	100.5
S6	2.70	99.6	0.18	116.9
S7	2.49	99.8	0.13	127.4
S8	2.82	99.3	0.19	111.1
S9	2.66	99.6	0.31	118.8
S10	2.71	99.1	0.23	115.0
S11	2.76	99.4	0.17	114.0
S12	2.65	98.9	0.29	117.0
S13	3.18	99.2	0.24	98.3
S14	2.82	99.5	0.29	111.8
S15	2.87	99.1	0.34	108.9
S16	2.82	99.3	0.19	111.1
Average	2.77	99.3	0.26	113.9

## Data Availability

The data are available from the corresponding author upon reasonable request.
